# Finite Element Analysis of Acetabulum Prosthesis' Lining Damage Zone with Different Implanting Angle

**DOI:** 10.1155/2023/9350474

**Published:** 2023-06-02

**Authors:** Yiqun Bian, Hao Wang, Anqi Huang

**Affiliations:** ^1^Liaocheng People's Hospital, China; ^2^Liaocheng Traditional Chinese Medicine Hospital, China

## Abstract

**Objective:**

Research the acetabular component's construction method of a three-dimensional finite element model in THA with different angles and study the influence of polyethylene liner wearing with finite element analysis.

**Methods:**

Build a model in the 3D modeling software system HyperMesh according to the artificial hip joint prosthesis' entities and data. Using a finite element analysis system, ABAQUS 6.11 reconstitute acetabular prosthesis after hip replacement joints under different implanting position angles. Simulation and load the joint load when sheet foot touchdown state. Calculate the plastic volume strain and fatigue fracture.

**Results:**

The two groups of combinations of abduction angle 50° vs. anteversion angle 10° and abduction angle 55° vs. anteversion angle 15° have been found to have relatively smaller interface plastic strain and fatigue fracture volume value (2.241 × 10^−7^ m^3^, 2.443 × 10^−7^ m^3^), respectively.

**Conclusion:**

The groups of combinations of abduction angle 50° vs. anteversion angle 10° have been found to have relatively smallest interface plastic strain and fatigue fracture volume value in the total hip arthroplasty.

## 1. Introduction

Total hip arthroplasty (THA) is currently the preferred treatment for serious hip problems. In other words, artificial hip prostheses are used to replace human hip implants and replace the original functions of joints, so as to achieve the goal of radical treatment of diseases [1–4]. A large number of long-term clinical follow-up results show that the acetabular prosthesis has a higher loosening rate and revision rate than the femoral lateral prosthesis, and the acetabular lining is considered to be the most vulnerable one. The joint stress can cause different degrees of plastic strain and long-term creep which is called the failure zone in the lining when the postoperative patients move after total hip replacement. The lining damage zone is different at different hip prosthesis placement angles.

In this project, the three-dimensional finite element model of an acetabular artificial prosthesis with different forward angles and abductor angles was first established. After loading, the fatigue fracture volume of the acetabular polyethylene liner was analyzed to reflect the long-term stress changes of the polyethylene lining after an operation. It provides theoretical guidance for acetabular prosthesis installation during operation and a theoretical basis for clinical application.

## 2. Materials and Methods

### 2.1. Main Experimental Equipment and Software

The following are the main experimental equipment and software: computer workstation (Intel Core I712700 5.0 GHz); memory (16GB DDR4); hard disk (4 TB 7200RPM); SATA3; 3D modeling software system (HyperMesh 14.0); and finite element analysis system (ABAQUS 6.11).

### 2.2. Establishment of Finite Element Model

According to the entity and design template of Chunli acetabular prosthesis (Figure 1), a 3D finite element model was established in the 3D modeling software HYPERMESH 14.0. Acetabular prosthesis with an inner diameter of 28 mm and corresponding femoral head were established, respectively. The thickness of the metal mortar cup is 4.6 mm, and the thickness of the polyethylene lining is 8 m (Figure 2).

### 2.3. Material Properties

So far, ultrahigh molecular weight polyethylene (UHMWPE) has been tested in clinical practice for more than 40 years as the material of choice for the acetabular prosthesis. However, the wear particles produced by UHMWPE bearing surface (especially 0.1 a 1.0 microns) activate macrophages in the tissue around the implant, release some active factors and inflammatory mediators, encourage osteoclast dissolving process of bone, dissolving the bone tissue around the implant bone, and lead to joint prosthesis loosening, thus affect the long-term effects of the joint replacement [5].

The UHMWPE has an elastic modulus of 1.4GPa, a Poisson's ratio of 0.3, and a yield strength of 14 MPa.The stress-strain curve is shown in Figure 3, adopting the elastic-plastic parameters proposed by Sun et al. [6].

The metal cup and femoral head are made of diamond chrome with an elastic modulus of 210 GPa and a Poisson's ratio of 0.3.

### 2.4. Meshing and Optimization

The established hip prosthesis model was imported into ABAQUS for analysis. The polyethylene lining is an elastoplastic deformation body, and the lining is divided into 43280 units by using four-node tetrahedral isoparametric elements. The metal cup and the femoral head are elastomers, which are 36320 and 23260 units, respectively. The contact algorithm is applied to the articular surface of the femoral head and lining, the back of the lining, and the metal socket cup. The specific shape of the unit is shown in Figure 4.

### 2.5. Boundary Conditions and Force Loading of Acetabular Prosthesis Calculated by Finite Element Method

Due to the influence of anatomical factors and human activities, the main force of the hip joint occurs on the coronal plane, so in the past, only static load loading on the coronal plane of the hip joint was carried out for mechanical analysis. In the coronal two-dimensional plane, the joint force was calculated according to the effective body weight at the hip joint, the body weight moment arm, the gluteus medius muscle pull, and the muscle force moment arm. In this experiment, the load of the hip joint under the condition of a single-foot landing in a loaded standing position was used to simulate the force of the hip joint in three-dimensional space and carry out the mechanical analysis. When standing at rest on one foot, about 81% of the body weight is borne by the hip joint. The resultant force on the joint passes through the center of the femoral head at an angle of about 16 degrees perpendicular to the ground. The resultant force on the acetabulum was converted into the acetabulum in three-dimensional space, and the inward, backward, and upward directions of the *X*, *Y*, and *Z* directions were positive, and the forces were *X* = 486 N; *Y* = 1468 N; *Z* = 848 N.

### 2.6. Parametric Modeling

A total of 25 different combinations can be obtained for different combinations of abduction angle and rake angle, and the models under the 25 combinations are not the same. For example, the establishment of one will consume a lot of time and energy. In this modeling process, the method of “parametric modeling” is adopted. Parametric modeling is to read the user's requirements (abduction angle, rake angle, and different combinations) by compiling corresponding programs and then to carry out procedural modeling according to the user's requirements. In this modeling process, ABAQUS user interaction program Python language was used to compile the corresponding modeling program and realize the program modeling.

## 3. Result

In this study, the failure zone volume was simulated when the acetabular opening forward Angle was 0°, 5°, 10°, 15°, 20°, and 25°, and the abduction Angle was 30°, 35°, 40°, 45°, 50°, and 55°.

Volume size and analysis cloud diagram of plastic strain failure zone at the interface of polyethylene lining.

The failure zone volume of polyethylene liner in the hip joint varies with different placement angles. A total of 25 combinations can be obtained for different combinations of the elongation angle and rake angle, corresponding to different failure zone size results (Table 1). With the change of abduction angle and rake angle, the volume of the failure zone also changes. The combination of the abduction angle of 50° and anteversion angle of 10° and the combination of the abduction angle of 55° and anteversion angle of 15° had the smallest volume of polyethylene liner failure zone, which were 2.443 × 10^−7^ m^3^ and 2.241 × 10^−7^ m^3^, respectively (Figure 5).

A comprehensive analysis of the failure zone volume of polyethylene lining shows that there is an interaction between the hip joint rake angle and abduction angle, which jointly affect the force of polyethylene. With the increase of abduction angle, the coverage area of the femoral head increased, and the volume of damage area decreased continuously. With the increase of the rake angle, the failure zone volume of the polyethylene liner becomes larger (Figure 6).

## 4. Discussion

### 4.1. Significance of Three-Dimensional Finite Element Analysis for Total Hip Arthroplasty

After more than 60 years of continuous improvement, THA has become a routine operation for the treatment of severe hip diseases, which can effectively relieve hip pain, improve hip function, restore joint stability, and improve hip deformity. However, the fatal defect of THA is its limited prosthesis life [6]. Prosthesis installation is an important factor causing prosthesis loosening and dislocation. The normal biomechanics of the body is changed after implant implantation, but it is difficult to observe and analyze by traditional research methods. This experiment attempted to establish a three-dimensional model of the prosthesis after total hip arthroplasty and the finite element mechanical analysis method to simulate the stress in the joint after the operation and the damage degree of the stress on the prosthesis lining material. It provides a new way for joint stress simulation and surgical evaluation analysis in the future.

### 4.2. Influence of Different Prosthesis Materials on Finite Element Analysis

Cobalt-chromium-molybdenum alloy, alumina ceramics, and zirconia ceramics are the main femoral head prosthesis materials used to match with polyethylene lining in total hip arthroplasty [7]. They have different elastic moduli and Poisson's ratios, but the elastic modulus and Poisson's ratio of femoral head prosthesis materials have no significant influence on contact stress. Therefore, the established test can well reflect the stress of femoral head prosthesis of different materials on polyethylene lining [8, 9]. However, various materials have different friction coefficients and will produce different friction rates when matched with UHMWPE acetabular prosthesis, resulting in different degrees of wear [10].

Related studies [11–17] reported that the annual wear rate of ceramic and polyethylene acetabular cups was significantly lower than that of metal and polyethylene. Solarino et al. [18] showed that metal femoral head prosthesis has poor antiwear performance on ultrahigh molecular weight polyethylene artificial hip joint, which is easy to cause osteolysis and loosening. Ceramic has good friction, wear, and lubrication properties on the ceramic artificial hip joint, and there is no wear particles and osteolysis after hip prosthesis replacement. The fourth-generation ceramic material has become the preferred femoral head prosthesis material for hip replacement due to its hard texture, biological inertia, and low friction coefficient [13, 19, 20]. Although the finite element analysis model in this experiment can reflect the stress of the femoral head with different materials on the lining, osteolysis caused by interfacial friction and its induced particles is not considered [21, 22].

This paper mainly studies the different lining failure zones caused by different prosthesis installation angles after THA. The conclusion is 50°of the abduction angle and 10° of the anteversion angle are the installation angles with the smallest volume (2.241 × 10^−7^ m^3^) in total hip arthroplasty. In this paper, it is considered that under the premise of the same prosthesis material and prosthesis design, the best prosthesis installation angle is the abduction angle of 50° and forward angle of 10°. However, the model established in this paper is only an ideal model and does not take into account the force exerted by the soft tissue around the joint. Besides the influence of the installation angle of the prosthesis, the service life of the prosthesis is also affected by other factors.

### 4.3. The Effect of Implant Angle on Prosthesis Survival

The survival rate of the acetabular prosthesis is affected by many factors, such as age, weight, and fixation method. Aseptic loosening of the acetabular prosthesis is one of the important reasons for surgical failure. Some long-term follow-up studies after hip replacement have found significant differences in long-term survival while short-term survival with the prosthesis is similar [23]. This follow-up result is consistent with microwear caused by stress concentration. Our study showed that different angles of the acetabular prosthesis can lead to stress concentration. Stress concentration can lead to extensive wear of the polyethylene lining, and worn polyethylene particles can induce an autoimmune response that leads to bone resorption and bone destruction at the bone-prosthesis interface, leading to aseptic loosening of the prosthesis. Severe misalignment of the acetabular prosthesis can also lead to limited joint movement, pain, and even dislocation of the hip. The correct installation Angle can reduce the wear of the polyethylene lining and reduce aseptic loosening, which plays a key role in prolonging the survival rate of the prosthesis.

## 5. Conclusion

Relatively small interfacial plastic strain and fatigue fracture volume values (2.241 × 10^−7^ m^3^ and 2.443 × 10^−7^ m^3^) were obtained by the combination of an abduction angle of 50° and forward inclination of 10° and abduction angle of 55° and forward inclination of 15°. In addition, the installation angle of the abduction angle of 50° and the forward inclination angle of 10° is less than that of the abduction angle of 55° and the forward inclination angle of 15°. The results of finite element analysis showed that the optimal angle of acetabular prosthesis installation in total hip arthroplasty should be an abduction angle of 50° and an anteversion angle of 10°.

## Figures and Tables

**Figure 1:** Chunli acetabular prosthesis.

**Figure 2:** Model of polyethylene lining and femur head.

**Figure 3:** Stress-stain curve of UHMWPE.

**Figure 4:** The established hip prosthesis model was imported into ABAQUS for analysis.

**Figure 5:** (a) Stress profile of polyethylene lining at 50° abduction and 10° forward inclination. (b) Stress profile of polyethylene lining at 45° abduction and 15° forward inclination.

**Figure 6:** (a) Polyethylene lining stress results in nephogram. (b) Polyethylene lining failure zone volume results in nephogram.

**Table 1:** Polyethylene lining failure zone volume results.

	Former angle 0°	Former angle 5°	Former angle 10°	Former angle 15°	Former angle 20°	Former angle 25°
Outreach angle 30°	9.025	8.510	7.250	9.055	9.340	8.511
Outreach angle 35°	6.461	5.771	6.500	7.197	7.780	7.933
Outreach angle 40°	5.109	6.306	6.554	5.880	4.871	4.005
Outreach angle 45°	5.302	3.233	8.262	3.144	4.338	5.837
Outreach angle 50°	3.542	4.550	2.241	4.883	4.066	4.494
Outreach angle 55°	3.801	3.411	2.872	2.443	3.164	4.967

Unit:^∗^10^−7^ m^3^.

## Data Availability

Data sharing is not applicable to this article as no datasets were generated or analyzed during the current study.
